The article "Hematologic Cancer Detection Using White Blood Cancerous Cells Empowered with Transfer Learning and Image Processing" was published in 2023. Journal: J Healthc Eng.

# Hematologic Cancer Detection Using White Blood Cancerous Cells Empowered with Transfer Learning and Image Processing

**DOI:** 10.1155/2023/1406545

**Published:** 2023-05-29

**Authors:** Muhammad Umar Nasir, Muhammad Farhan Khan, Muhammad Adnan Khan, Muhammad Zubair, Sagheer Abbas, Meshal Alharbi, Md Akhtaruzzaman

**Affiliations:** ^1^Department of Computer Science, Bahria University, Lahore Campus, Lahore 54000, Pakistan; ^2^Department of Forensic Sciences, University of Health Sciences, Lahore 54000, Pakistan; ^3^Riphah School of Computing and Innovation, Faculty of Computing, Riphah International University, Lahore Campus, Lahore 54000, Pakistan; ^4^School of Information Technology, Skyline University College, University City Sharjah, Sharjah, UAE; ^5^Faculty of Computing, Riphah International University, Islamabad 45000, Pakistan; ^6^School of Computer Science, National College of Business Administration & Economics, Lahore 54000, Pakistan; ^7^Department of Computer Science, College of Computer Engineering and Sciences, Prince Sattam Bin Abdulaziz University, Alkharjb 11942, Saudi Arabia; ^8^Department of Computer Science and Engineering, Aisan University of Bangladesh, Ashulia, Dhaka-1230, Bangladesh

## Abstract

Lymphoma and leukemia are fatal syndromes of cancer that cause other diseases and affect all types of age groups including male and female, and disastrous and fatal blood cancer causes an increased savvier death ratio. Both lymphoma and leukemia are associated with the damage and rise of immature lymphocytes, monocytes, neutrophils, and eosinophil cells. So, in the health sector, the early prediction and treatment of blood cancer is a major issue for survival rates. Nowadays, there are various manual techniques to analyze and predict blood cancer using the microscopic medical reports of white blood cell images, which is very steady for prediction and causes a major ratio of deaths. Manual prediction and analysis of eosinophils, lymphocytes, monocytes, and neutrophils are very difficult and time-consuming. In previous studies, they used numerous deep learning and machine learning techniques to predict blood cancer, but there are still some limitations in these studies. So, in this article, we propose a model of deep learning empowered with transfer learning and indulge in image processing techniques to improve the prediction results. The proposed transfer learning model empowered with image processing incorporates different levels of prediction, analysis, and learning procedures and employs different learning criteria like learning rate and epochs. The proposed model used numerous transfer learning models with varying parameters for each model and cloud techniques to choose the best prediction model, and the proposed model used an extensive set of performance techniques and procedures to predict the white blood cells which cause cancer to incorporate image processing techniques. So, after extensive procedures of AlexNet, MobileNet, and ResNet with both image processing and without image processing techniques with numerous learning criteria, the stochastic gradient descent momentum incorporated with AlexNet is outperformed with the highest prediction accuracy of 97.3% and the misclassification rate is 2.7% with image processing technique. The proposed model gives good results and can be applied for smart diagnosing of blood cancer using eosinophils, lymphocytes, monocytes, and neutrophils.

The article "Hematologic Cancer Detection Using White Blood Cancerous Cells Empowered with Transfer Learning and Image Processing" was published in 2023. Journal: J Healthc Eng.

## 1. Introduction

Leukemia and lymphoma are the most frequent kinds of blood cancer in people of all ages, particularly young people. This abnormal situation is induced by red blood cell proliferation and immature growth, which can harm red blood cells, bone marrow, and the immune system [1]. Leukemia accounts for more than 3.5% of new cancer cases in the United States, with over 50,000 new cases diagnosed in 2018 [2]. Cancerous lymphoblasts in the blood travel to other organs, including the heart, brain, lungs, and arteries, before spreading to important tissues throughout the body. Red blood cells are normally in charge of transporting oxygen from the heart to all organs. They make up half of the total blood volume. White blood cells, on the other hand, serve an important role in the human immune system, serving as the first line of protection against a variety of diseases and disorders [3]. As a result, accurately identifying these white blood cells is crucial in understanding the symptoms of the problem. Their categorization is determined by their cytoplasmic composition. Changes in lymphocytes, a kind of white blood cell, cause acute lymphoblastic leukemia [4]. Acute or chronic leukemia are the two types of leukemia. Without treatment, the typical recovery period for acute myeloid leukemia is roughly three months; however, the time of appearance of chronic leukemia is longer than that of acute leukemia. Chronic lymphoblastic leukemia is the most common kind of acute leukemia, accounting for around 25% of all juvenile malignancies [5, 6]. Early detection of leukemia and lymphoma has always been difficult for researchers, clinicians, and hematologists. Leukemia symptoms include enlarged lymph nodes, paleness, fever, and weight loss, although these symptoms can also be caused by other diseases [7]. Because of the moderate nature of the symptoms, diagnosing leukemia and lymphoma in its early stages is challenging. PBS microscopic assessment is the most often used leukemia and lymphoma diagnostic approach, while the gold standard for leukemia and lymphoma diagnosis only entails obtaining and analyzing white blood cell samples [8]. Several research have utilized machine learning and deep learning and machine diagnostics approaches to laboratory image processing during the last two decades in the hopes of pushing the boundaries of late diagnosis of leukemia and lymphoma and establishing their subtypes [9]. In this research, blood smear pictures were evaluated to diagnose, distinguish, and count cells in distinct kinds of leukemia and lymphoma [10].

The article "Hematologic Cancer Detection Using White Blood Cancerous Cells Empowered with Transfer Learning and Image Processing" was published in 2023. Journal: J Healthc Eng.

Deep learning is a famous artificial intelligence area that comprises algorithms and statistical associations. It has quickly permeated the field of clinical research. Deep learning allows you to teach machines without prior skills and discover your knowledge. The application of these technologies to medical data processing achieved outstanding results and was especially beneficial in disease detection [11]. Deep learning techniques, according to studies, significantly help [12] the complex medical decision-making processes in medical image processing [13] by extracting and then analyzing characteristics from these pictures [14]. As the number of medical diagnostic instruments increased and a considerable volume of high-quality data was created, there was an urgent demand for more powerful data processing technologies. Conventional data analysis methods were incapable of analyzing such massive volumes of data or identifying data trends.

The proposed study employs deep learning procedures driven by transfer learning and image processing to overcome the limitations of earlier investigations. The following are the study's significant contributions:

- The proposed study used transfer learning incorporated with various algorithms for better prediction results
- The proposed study used a generic approach and comparative analysis techniques have shown that the proposed study of deep learning empowered with transfer learning with image processing outperformed using the white blood cell dataset
- For enhanced results, the proposed study uses image processing practices
- Private data cloud techniques are used for data and model security
- For performance evaluation, the proposed model used numerous performance matrices

## 2. Literature Review

Image analysis of contaminated blood cells is frequently separated into four stages: preparation, extraction, feature engineering, and classification. Extensive research has been conducted on numerous types of cancer, including leukemia and lymphoma. Zhang et al. proposed a convolutional neural network (CNN) model for the nonsegmented direct sorting of tissue samples into healthy and sick cells [15]. To categorize distinct kinds of white blood cells in the body, Zhao et al. offered machine-learning approaches such as CNN, support vector machine (SVM), random forest, and others [16].

The article "Hematologic Cancer Detection Using White Blood Cancerous Cells Empowered with Transfer Learning and Image Processing" was published in 2023. Journal: J Healthc Eng.

The relative white blood cell ratio is used to determine the morphology of leukemia and lymphoma. Deep learning-based computational analysis has shown promise as a diagnostic technique for heterogeneous white blood cell count. Deep learning was demonstrated by Choi et al. [17] and Qin et al. [18] to categorize white blood cells at numerous stages of maturation, laying the foundation for a deep learning-based diagnosis of leukemia and lymphoma; however, these research findings had constraints due to a shortage of cell types and poor sensitivity, respectively, and classification was usually done using precompiled images rather than raw clinical images. The white blood cell disparity ratio for myeloid analysis is an important use of transfer learning that still requires improvement.

Karthikeyan and Poornima [19] described a novel method for segmenting and classifying acute myeloid and lymphomas that were preprocessed using histogram equalization and median filtering. Two techniques for lymphocyte segmentation were compared: clustering algorithm and k-mean. For lymphocyte segmentation, fuzzy c-means clustering beats k-means clustering. After that, the support vector machine was utilized to separate normal and blast cells. MoradiAmin et al. [20] separated background lymphocytes using widespread pooling of C medium to increase the identification of acute lymphocytic leukemia cells. Following the extraction of diverse shape-based data, they used hierarchical clustering to minimize the number of parameters before providing them to assist the SVM classifier for normal and popping cell categorization.

The authors of the study employed computer vision techniques to overcome the difficulties of manual counting. In this situation, the picture has been preprocessed to remove the chance of distortion, and the proportion of white blood cells to red blood cells has been determined to determine if the image is normal or abnormal for detecting Salihah et al. [21]. Horie et al. [22] proved the diagnostic effectiveness of deep learning approaches such as CNN for esophagitis, including melanoma and adenocarcinoma, with a sensitivity of 98%.

The authors [23] developed a CNN model for leukemia prediction that featured three key steps: CNN comparison stretching and edge extraction, followed by transfer learning depth feature extraction. In [24], authors developed a method for distinguishing tainted pictures from healthy ones that uses a convolutional neural network. Furthermore, the clustering method using the EM approach is utilized to compute the rate of infection spread thus far. The study [25] proposed computer-aided diagnostic methods for leukemia cancer classification using an ensembled SVM learning approach. The authors proposed a supervised machine learning approach to identify blood cancer and then categorise them using a fully integrated network [26].

The article "Hematologic Cancer Detection Using White Blood Cancerous Cells Empowered with Transfer Learning and Image Processing" was published in 2023. Journal: J Healthc Eng.

The study offered classification models for distinguishing microscopic pictures of blood from leukemia and lymphoma patients from those who were not [27]. A pretrained CNN named AlexNet, as well as numerous additional classifiers, are utilized to extract the features. In comparison to other classifiers, the support vector machine fared better in tests. In the second model, AlexNet is used for extraction and classification only when the results demonstrate that it outperforms other models on various performance criteria.

The authors of this study [28] presented a computational method for detecting acute leukemia and lymphoma. To begin, focusing was applied to digital microscope pictures to decrease noise and blurring. Color, form, texture, and statistics were identified and classed as benign or malignant. Classification models based on K-nearest neighbors and naive Bayes were utilized. Experiments with sixty blood analyzers proved the effectiveness of the K-nearest neighbor (KNN), which had a 92.8% accuracy rate.

The authors of this study [29] created a mechanism for categorizing acute myelogenous leukemia cells into subgroups. Initially, cells were segmented using a color k-means technique. Following that, six statistical characteristics were retrieved and fed into a multiclass SVM classifier. The data yielded a maximum aiming accuracy of 87% and a maximum accuracy of 92.9%.

According to the study [30], a three-tier approach including extracting features, coding, and categorization is recommended. The goal of this approach was to evaluate whether or not a patient has leukemia or lymphoma based on a picture of a sample of blood from a particular patient. A thick structurally complex transformation was used in feature extraction. At the encoding layer, the size of the recovered feature vectors was lowered. Finally, a multiclass support vector machine classifier was used to do the classification. Experiments with four hundred samples resulted in an accuracy of 79.38%.

The study [31] established a classification system for acute myelogenous leukemia that segments grains using contour and k-signature methods. Then, utilizing the morphology, characteristics such as cell volume, cell color, and so on were retrieved. Studies on a dataset of one hundred pictures found that the SVM classifier had up to 92% classification accuracy.

The article "Hematologic Cancer Detection Using White Blood Cancerous Cells Empowered with Transfer Learning and Image Processing" was published in 2023. Journal: J Healthc Eng.

The study [32] described an automated microscopic image-based technique for diagnosing leukemia and lymphoma. The technique begins by reducing noise and blur during preprocessing. The white blood cells were then separated using the k-means and Zack algorithms. Following that, chromatic, statistical, geometric, and textural elements were restored. Finally, to distinguish between healthy and unhealthy images, an SVM classifier was utilized. Trials on a dataset of twenty-seven pictures revealed a 93.57% classification accuracy.

The research [33] created a categorization system for three forms of acute myeloid leukemia and acute multiple myeloma leukemia and acute lymphocytic leukemia. Twelve characteristics were extracted by hand from picture samples. Finally, for classification, a K-nearest neighbor predictor was applied. Experiments using a sample of 350 photos yielded 86% reliability. The authors [34] developed a five-characteristic method for acute myelogenous leukemia categorization that improved picture contrast. An SVM classifier was used to categorize the data. Experiments with 51 photos provided a categorization accuracy of 93.5%.

To categorize acute lymphocytic leukemia and its subtypes, the authors [35] recommended using a CNN network termed a convolutional network. A dataset of 373 pictures was utilized for the evaluation, and an accuracy of 80% was reached. Experiments confirmed this method's superiority over a range of earlier techniques. The authors [36] used numerous deep learning approaches to predict blood cancer cells including CNN and SVM and they achieved 97.04% prediction accuracy.

Previous research on the prediction of blood cancer utilizing white blood cells using machine learning and deep learning had significant drawbacks. The limitations of prior investigations are shown in Table 1.

As Table 1 depicts the summary of all previous research that predicted blood cancer using machine learning, deep learning, and transfer learning techniques, every study has its own limitations. So, this study has the advantage of coping with all these limitations wisely during blood cancer prediction.

## 3. Materials and Methods

Figure 1 depicts an overview of the suggested approach for predicting blood cancer using transfer learning-enabled malignant white blood cells. The proposed process begins with data input from several hospital sources. After collecting all white blood cell (WBC) samples, data augmentation techniques were used to overcome the challenges of mining data samples for WBC classes. The proposed methodology depicts four major steps in the whole prediction process for blood cancer. In the first phase, the proposed framework collects data from the hospital, preprocessed blood samples, divides all preprocessed samples into training testing sample ratios, and stores these split samples in private for easy access at any step. The training phase imports training data samples from the private cloud and trains the AlexNet, ResNet, and MobileNet algorithms with stochastic gradient descent (SGD) with momentum, adaptive momentum estimation, and signal propagation algorithms using squares of the root. After training all algorithms of AlexNet, ResNet, and MobileNet, applying learning criteria techniques, if the learning criteria match the proposed framework expectations, then the trained model is stored separately on each algorithm's private cloud. If the proposed model does not meet the learning criteria then apply image processing techniques such as histogram equalization and again train the model and check the learning criteria.

The article "Hematologic Cancer Detection Using White Blood Cancerous Cells Empowered with Transfer Learning and Image Processing" was published in 2023. Journal: J Healthc Eng.

In the third phase, choose the semi-best-trained algorithms from all private clouds and store them in another private cloud for the further testing processes. In the last phase, which is known as the testing phase, import blood samples from the cloud, import the best-performed trained model from the model secluded, and apply the testing process to predict the cancerous white blood cells. Finally, the proposed framework used numerous statistical matrices [37–43], e.g., classification accuracy (CA), negative predicted value (NPV), sensitivity, specificity, f1-score, miss-classification rate (MCR), positive predicted value (PPV), likelihood positive ratio (LPR), false negative rate (FNR), likelihood negative ratio (LNR), false positive rate (FPR), and Fowlkes Mallows index (FMI), all statistical matrix equations are given as follows:

(1) $$\begin{array}{c} \partial_{i}=\frac{{ℵ}_{i}}{\zeta_{i}}\text{.} \end{array}$$

∴*ζ* for true class and ℵ is for the predicted class:

(2) $$\begin{array}{c} \chi_{i}=\overset{3}{\underset{j=1}{\sum }}\left(\frac{{ℵ}_{i}}{\zeta_{j\neq i}}\right)\text{,}\\ \varsigma_{i}=\overset{3}{\underset{j=1}{\sum }}\left(\frac{{ℵ}_{j\neq i}}{\zeta_{i}}\right)\text{,}\\ \varrho_{i}=\overset{3}{\underset{j=1}{\sum }}\left(\frac{{ℵ}_{j\neq i}}{\zeta_{j\neq i}}\right)\text{,}\\ CA=\frac{{ℵ}_{i}/\zeta_{i}+\sum_{j=1}^{3}\left({ℵ}_{i}/\zeta_{j\neq i}\right)}{{ℵ}_{i}/\zeta_{i}+\sum_{j=1}^{3}\left({ℵ}_{i}/\zeta_{j\neq i}\right)+\sum_{j=1}^{3}\left({ℵ}_{j\neq i}/\zeta_{i}\right)+\sum_{j=1}^{3}\left({ℵ}_{j\neq i}/\zeta_{j\neq i}\right)}*100\text{,}\\ CMR=100-\left(\frac{{ℵ}_{i}/\zeta_{i}+\sum_{j=1}^{3}\left({ℵ}_{i}/\zeta_{j\neq i}\right)}{{ℵ}_{i}/\zeta_{i}+\sum_{j=1}^{3}\left({ℵ}_{i}/\zeta_{j\neq i}\right)+\sum_{j=1}^{3}\left({ℵ}_{j\neq i}/\zeta_{i}\right)+\sum_{j=1}^{3}\left({ℵ}_{j\neq i}/\zeta_{j\neq i}\right)}*100\right)\text{,}\\ sensitivity=\frac{{ℵ}_{i}/\zeta_{i}}{{ℵ}_{i}/\zeta_{i}+\sum_{j=1}^{3}\left({ℵ}_{j\neq i}/\zeta_{j\neq i}\right)}*100\text{,}\\ specificity=\frac{\overset{3}{\underset{j=1}{\sum }}\left({ℵ}_{i}/\zeta_{j\neq i}\right)}{\overset{3}{\underset{j=1}{\sum }}\left({ℵ}_{i}/\zeta_{j\neq i}\right)+\overset{3}{\underset{j=1}{\sum }}\left({ℵ}_{j\neq i}/\zeta_{i}\right)}*100\text{,}\\ F1-score=\frac{2\;{ℵ}_{i}/\zeta_{i}}{2\;{ℵ}_{i}/\zeta_{i}+\sum_{j=1}^{3}\left({ℵ}_{j\neq i}/\zeta_{i}\right)+\overset{3}{\underset{j=1}{\sum }}\left({ℵ}_{j\neq i}/\zeta_{j\neq i}\right)}*100\text{,}\\ PPV=\frac{{ℵ}_{i}/\zeta_{i}}{{ℵ}_{i}/\zeta_{i}+\sum_{j=1}^{3}\left({ℵ}_{j\neq i}/\zeta_{i}\right)}*100\text{,}\\ NPV=\frac{\overset{3}{\underset{j=1}{\sum }}\left({ℵ}_{i}/\zeta_{j\neq i}\right)}{\overset{3}{\underset{j=1}{\sum }}\left({ℵ}_{i}/\zeta_{j\neq i}\right)+\overset{3}{\underset{j=1}{\sum }}\left({ℵ}_{j\neq i}/\zeta_{j\neq i}\right)}*100\text{,}\\ FPR=100-\left(\frac{\overset{3}{\underset{j=1}{\sum }}\left({ℵ}_{i}/\zeta_{j\neq i}\right)}{\overset{3}{\underset{j=1}{\sum }}\left({ℵ}_{i}/\zeta_{j\neq i}\right)+\overset{3}{\underset{j=1}{\sum }}\left({ℵ}_{j\neq i}/\zeta_{i}\right)}*100\right)\text{,}\\ FNR=100-\left(\frac{{ℵ}_{i}/\zeta_{i}}{{ℵ}_{i}/\zeta_{i}+\sum_{j=1}^{3}\left({ℵ}_{j\neq i}/\zeta_{j\neq i}\right)}*100\right)\text{,}\\ LPR=\frac{{ℵ}_{i}/\zeta_{i}/{ℵ}_{i}/\zeta_{i}+\sum_{j=1}^{3}\left({ℵ}_{j\neq i}/\zeta_{j\neq i}\right)*100}{100-\left(\overset{3}{\underset{j=1}{\sum }}\left({ℵ}_{i}/\zeta_{j\neq i}\right)/\overset{3}{\underset{j=1}{\sum }}\left({ℵ}_{i}/\zeta_{j\neq i}\right)+\overset{3}{\underset{j=1}{\sum }}\left({ℵ}_{j\neq i}/\zeta_{i}\right)*100\right)}\text{,}\\ LNR=\frac{100-\left({ℵ}_{i}/\zeta_{i}/{ℵ}_{i}/\zeta_{i}+\sum_{j=1}^{3}\left({ℵ}_{j\neq i}/\zeta_{j\neq i}\right)*100\right)}{\overset{3}{\underset{j=1}{\sum }}\left({ℵ}_{i}/\zeta_{j\neq i}\right)/\overset{3}{\underset{j=1}{\sum }}\left({ℵ}_{i}/\zeta_{j\neq i}\right)+\overset{3}{\underset{j=1}{\sum }}\left({ℵ}_{j\neq i}/\zeta_{i}\right)*100}\text{,}\\ FMI=\sqrt{\left(\frac{{ℵ}_{i}/\zeta_{i}}{{ℵ}_{i}/\zeta_{i}+\sum_{j=1}^{3}\left({ℵ}_{j\neq i}/\zeta_{j\neq i}\right)}*100\right)*\left(\frac{{ℵ}_{i}/\zeta_{i}}{{ℵ}_{i}/\zeta_{i}+\sum_{j=1}^{3}\left({ℵ}_{j\neq i}/\zeta_{i}\right)}*100\right)}\text{.} \end{array}$$

The descriptive algorithm of the proposed study for blood cancer prognostication utilizing transfer learning-enhanced white blood cells is shown in Table 2. It represents the specifics of the proposed framework's complete procedure.

The article "Hematologic Cancer Detection Using White Blood Cancerous Cells Empowered with Transfer Learning and Image Processing" was published in 2023. Journal: J Healthc Eng.

### 3.1. Dataset

In this proposed study, the dataset is acquired from the online source Ghaderzadeh et al. [43]. The dataset consists of four classes named eosinophils, lymphocytes, monocytes, and neutrophils. Machine learning algorithms are highly data hungry [44].

The proposed framework dataset consists of 10,000 instances, and each class instance consists of almost 2,500 blood samples.  Figure 2 shows the sample data instance of each blood sample class.

## 4. Image Processing

To overcome the classification accuracy deficiency problem, the proposed framework uses the image processing technique e-g histogram equalization to enhance the quality of blood samples. With the help of histogram equalization, as shown in Figures 3 and 4, the proposed framework enhances the contrast and intensity of pixels in blood samples. Equation (3) represents the distribution function of histogram equalization.

(3) $$\begin{array}{c} {DF}_{y}\left(m\right)=\overset{m}{\underset{n=0}{\sum }}\rho_{y\;\left(y=n\right)}\text{.} \end{array}$$

## 5. Simulation Results and Discussion

In this article, transfer learning has been used for the prediction of blood cancer empowered with eosinophils, lymphocytes, monocytes, and neutrophils incorporated into the blood cell dataset [45]. For simulation purposes to train and test the data sample, the proposed model used a MacBook Pro 2017, 16 giga byte random access memory, and Core i5 with a 512 Giga byte solid state drive. The proposed framework divided the dataset into 70% and 30% blood cells for training and testing, respectively. To remove the different anomalies in the dataset, different pre-processing techniques have been implemented. Numerous transfer learning algorithms have been used to train the models and test the data samples. Different phases of training and testing have been discussed and elaborated on in this article. To measure the performance of all trained models and test results, the proposed framework used statistical performance parameters, and all parameters' equations are mentioned above in the methodology section.

Figure 5 shows the training progress of SGD with momentum using AlexNet without image processing. To train this model, the proposed model set a learning rate of 0.001, 100 epochs, and 58 iterations per epoch. The proposed framework of this training model has a lot of distortion and does not converge until the last epoch; all this distortion happens due to the contrast and pixels unbalancing in the data samples. So, stochastic gradient descent with momentum achieves 75.78% of CA and 24.22% MCR.

Figure 6 shows the training progress of the adaptive momentum association using AlexNet without image processing. To train this model, the proposed study set a learning rate of 0.001, 100 epochs, and 58 iterations per epoch. The proposed framework of this training model has a lot of distortion and does not converge till the last epoch; all this distortion happens due to the contrast and pixels unbalancing in data samples. So, adaptive momentum association achieves 86.72% and 13.28% of classification accuracy and miss-classification rate, respectively.

The article "Hematologic Cancer Detection Using White Blood Cancerous Cells Empowered with Transfer Learning and Image Processing" was published in 2023. Journal: J Healthc Eng.

Figure 7 shows the training progress of root mean square (RMS) propagation using AlexNet without image processing. To train this model, the proposed study set a learning rate of 0.001, 100 epochs, and 58 iterations per epoch. The proposed framework of this training model has a lot of distortion and does not converge till the last epoch; all this distortion happens due to the contrast and pixels unbalancing in the data samples. So, root means square propagation achieves 75.78% of CA and 24.22% MCR.

Figure 8 shows the training progress of SGD with momentum using MobileNet without image processing. To train this model, the proposed study set a learning rate of 0.001, 100 epochs, and 58 iterations per epoch. The proposed framework of this training model has a lot of distortion and does not converge till the last epoch; all this distortion happens due to the contrast and pixel unbalancing in the data samples. So, stochastic gradient descent with momentum achieves 75.00% and 25.00% of CA and MCR, respectively.

Figure 9 shows the training progress of adaptive momentum association using MobileNet without image processing. To train this model, the proposed framework set a learning rate of 0.001, 100 epochs, and 58 iterations per epoch. The proposed framework of this training model has a lot of distortion and does not converge till the last epoch; all this distortion happens due to the contrast and pixels unbalancing in the data samples. So, adaptive momentum association achieves 82.03% of classification accuracy and 17.97% miss-classification rate, respectively.

Figure 10 shows the training progress of RMS propagation using MobileNet without image processing. To train this model, the proposed study set a learning rate of 0.001, 100 epochs, and 58 iterations per epoch. The proposed framework of this training model has a lot of distortion and does not converge till the last epoch; all this distortion happens due to the contrast and pixels unbalancing in the data samples. So, root means square propagation achieves 75.00% and 25.00% of CA and MCR, respectively.

Figure 11 shows the training progress of SGD with momentum using ResNet without image processing. To train this model, the proposed study set a learning rate of 0.001, 100 epochs, and 58 iterations per epoch. The proposed framework of this training model has a lot of distortion and does not converge till the last epoch; all this distortion happens due to the contrast and pixels unbalancing in the data samples. So, stochastic gradient descent with momentum achieves 87.50% of classification accuracy and 12.50% miss-classification rate, respectively.

The article "Hematologic Cancer Detection Using White Blood Cancerous Cells Empowered with Transfer Learning and Image Processing" was published in 2023. Journal: J Healthc Eng.

Figure 12 shows the training progress of adaptive momentum association using ResNet without image processing. To train this model, the proposed study set a learning rate of 0.001, 100 epochs, and 58 iterations per epoch. The proposed framework of this training model has a lot of distortion and does not converge till the last epoch, all this distortion happens due to the contrast and pixels unbalancing in the data samples. So, adaptive momentum association achieves 74.22% and 25.78% of classification accuracy and miss-classification rate respectively.

Figure 13 shows the training progress of RMS propagation using ResNet without image processing. To train this model, the proposed study set a learning rate of 0.001, 100 epochs, and 58 iterations per epoch. The proposed framework of this training model has a lot of distortion and does not converge till the last epoch; all this distortion happens due to the contrast and pixels unbalancing in the data samples. So, root means square propagation achieves 71.09% of classification accuracy and 28.91% miss-classification rate, respectively.

Table 3 shows the training results of AlexNet models after image processing; all models tune on 5800 iterations, a 0.001 learning rate, and 100 epochs. So, the stochastic gradient descent moment outperformed the supra each training model and achieves 99.2% of classification accuracy and 0.8% miss-classification rate, respectively.

Figure 14 shows the training progress of SGD moments using AlexNet after image processing. To train this model, the proposed study set a learning rate of 0.001, 100 epochs, and 58 iterations per epoch. The proposed framework of this training model converges before 90 epochs and gives the highest training results.

Table 4 shows the training results of ResNet models after image processing; all models tune on 5800 iterations, a 0.001 learning rate, and 100 epochs. So, RMSPROP outperformed all models and achieves a 69.53% and 30.47% of classification accuracy and miss-classification rate, respectively.

Table 5 shows the training results of MobileNet models after image processing; all models tune on 5800 iterations, a 0.001 learning rate, and 100 epochs. So, RMSPROP outperformed all models and achieves a 73.44% and 26.56% of classification accuracy and miss-classification rate, respectively.

The article "Hematologic Cancer Detection Using White Blood Cancerous Cells Empowered with Transfer Learning and Image Processing" was published in 2023. Journal: J Healthc Eng.

Table 6 shows the test simulation of AlexNet models after image processing. The proposed framework finds that SGDM performs very well as compared with other models. SGDM predicted 719 lymphocyte cancerous cells correctly, 742 monocyte cancerous cells, and 716 neutrophil cancerous cells correctly. SGDM achieves 97.3%, 2.7% of classification accuracy, and miss-classification rate, respectively. ADAM predicted 674 lymphocyte cancerous cells correctly, 703 monocyte cancerous cells, and 720 neutrophil cancerous cells correctly. ADAM achieves 93.7% of classification accuracy, 6.3% of classification accuracy, and a miss-classification rate, respectively. RMSPROP predicted 714 lymphocyte cancerous cells correctly, 680 monocyte cancerous cells, and 692 neutrophil cancerous cells correctly. RMSPROP achieves 93.2%, 6.8% of classification accuracy, and a miss-classification rate, respectively.

Table 7 shows the test simulation of MobileNet models after image processing. The proposed framework finds that RMSPROP performs very well as compared with other models. RMSPROP predicted 729 lymphocyte cancerous cells correctly, 559 monocyte cancerous cells, and 159 neutrophil cancerous cells correctly. RMSPROP achieves 64.9% and 35.1% of classification accuracy and miss-classification rate, respectively. ADAM predicted 676 lymphocyte cancerous cells correctly, 339 monocyte cancerous cells, and 390 neutrophil cancerous cells. ADAM achieves 63.0% of classification accuracy and 37.0% miss-classification rate, respectively. SGDM predicted 678 lymphocyte cancerous cells correctly, 284 monocyte cancerous cells, and 388 neutrophil cancerous cells correctly. SGDM achieves 60.5% of classification accuracy and 39.5% miss-classification rate, respectively.

Table 8 shows the test simulation of MobileNet models after image processing. The proposed framework finds that ADAM performs very well as compared with other models. ADAM predicted 736 lymphocyte cancerous cells correctly, 319 monocyte cancerous cells, and 428 neutrophil cancerous cells. ADAM achieves 66.5%, and 33.5% of classification accuracy and miss-classification rate respectively. RMSPROP predicted 728 lymphocyte cancerous cells correctly, 608 monocyte cancerous cells, and 128 neutrophil cancerous cells. RMSPROP achieves 65.6%, and 34.4% of classification accuracy and miss-classification rate respectively. SGDM predicted 717 lymphocyte cancerous cells correctly, 409 monocyte cancerous cells, and 352 neutrophil cancerous cells correctly. SGDM achieves 66.2% of classification accuracy and 33.8% miss-classification rate, respectively.

The article "Hematologic Cancer Detection Using White Blood Cancerous Cells Empowered with Transfer Learning and Image Processing" was published in 2023. Journal: J Healthc Eng.

Table 9 shows the statistical matrix results of blood cancer prediction after image processing. These results depict that the SGDM of AlexNet outperthiformed all models and achieves 97.3% classification accuracy and a 2.7% miss-classification rate. SGDM of MobileNet performed below the performance line and achieved 60.5% classification accuracy and a 39.5% miss-classification rate.

Table 10 shows the testing results of all models, and SGDM of AlexNet is outperformed as compared with other models and achieves 78.6% classification accuracy, 21.4% of classification accuracy, and miss-classification rate, respectively. But when the proposed framework compared these results with the results of after-image processing, the results of the proposed model after-image processing performed well as compared with these. The proposed framework performed outstandingly as compared with the previous studies.

Table 11 depicts the descriptive comparative analysis of this study with previous work, so the analysis depicts Pansombut et al. [35] achieved 80% classification accuracy, 20% miss-classification rate empowered with the CNN model on publicly available image blood samples, Madhukar et al. [34] achieved 93.5% classification accuracy, 6.5% miss-classification rate empowered with an SVM classifier on publicly available image blood samples. Supardi et al. [33] achieved 86% classification accuracy and a 14% miss-classification rate empowered with the KNN model on publicly available image blood samples, Mishra and Patel [32] achieved 93.57% classification accuracy, 6.53% miss-classification rate empowered with SVM classifier on publicly available image blood samples. Laosai and Chamnongthai [31] achieved 92% classification accuracy and an 18% miss-classification rate empowered with the SVM model on publicly available image blood samples. Faivdullah et al. [30] achieved 79.38% classification accuracy, 20.72% miss-classification rate empowered with the SVM model on publicly available feature-based blood samples. Setiawan et al. [29] achieved 87% classification accuracy and 13% miss-classification rate empowered with SVM and K-means model on publicly available image blood samples. Kumar et al. [28] achieved 92.8% classification accuracy and 17.2% miss-classification rate empowered with CNN, Naïve Bayes, and KNN models on publicly available image blood samples. Loey et al. [27] achieved 94.3% classification accuracy and 5.7% miss-classification rate empowered with CNN and AlexNet models on publicly available image blood samples, on the other side, the proposed study achieved the highest classification accuracy of 97.3% and a 2.7% of miss-classification rate because the proposed framework used image processing techniques empowered with various transfer learning algorithms.

The article "Hematologic Cancer Detection Using White Blood Cancerous Cells Empowered with Transfer Learning and Image Processing" was published in 2023. Journal: J Healthc Eng.

## 6. Conclusion and Future Work

The early detection of blood cancer using white blood cells can help meritoriously in its cure. The study's proposed framework consists of three transfer learning models AlexNet, MobileNet, and ResNet empowered with SGDM, ADAM, and RMSPROP. The proposed framework applies all transfer learning models with varying learning rates effectively to white blood cancerous cells for early classification. To enhance the results, the proposed study used image processing techniques incorporating transfer learning and achieved the highest CA of 97.3% and 2.7% MCR. All experiments in the proposed study are comprehensively explained with respect to every model training and testing phase. This study helps health 5.0 to predict blood cancer in its early stages for early treatment. Furthermore, in the future, federated machine learning using the fed average technique will play a major role in better early prediction of blood cancer empowered with fuzzed machine learning and deep learning techniques will also apply more statistical techniques such as ANOVA and Chi-Square.

## Figures and Tables

**Figure 1:** The proposed methodology for prediction of blood cancer using white blood cells empowered with transfer learning (this shows the research methodology of the current study, the overall process how data is fetching, training, and testing).

**Figure 2:** Data samples of all white blood cancerous cells (this shows some data samples for the easiness of the reader, learner, and other researchers). (a) Eosinophil. (b) Lymphocyte. (c) Monocyte. (d) Neutrophil.

**Figure 3:** Blood cell samples before image processing (this depicts the results of data samples before image preprocessing in the form of histogram equalization).

**Figure 4:** Blood cell samples after image processing (this depicts the results of data samples after image preprocessing in the form of histogram equalization).

**Figure 5:** Training progress of SGDM and AlexNet without image processing (this depicts the training progress of SGDM and AlexNet before the image processing phase and shows fluctuation).

**Figure 6:** Training progress of Adam of AlexNet without image processing (this depicts the training progress of adam and AlexNet before the image processing phase and shows fluctuation).

**Figure 7:** Training progress of RMSPROP of AlexNet without image processing (this depicts the training progress of RMSPROP and AlexNet before the image processing phase and shows fluctuation).

**Figure 8:** Training progress of SGDM of the mobile net without image processing (this depicts the training progress of SGDM and MobileNet before the image processing phase and shows fluctuation).

The article "Hematologic Cancer Detection Using White Blood Cancerous Cells Empowered with Transfer Learning and Image Processing" was published in 2023. Journal: J Healthc Eng.

**Figure 9:** Training progress of adam on the mobile net without image processing (this depicts the training progress of adam and MobileNet before the image processing phase and shows fluctuation).

**Figure 10:** Training progress of RMSPROP of the mobile net without image processing (this depicts the training progress of RMSPROP and MobileNet before the image processing phase and shows fluctuation).

**Figure 11:** Training progress of SGDM of ResNet without image processing (this depicts the training progress of SGDM and ResNet before the image processing phase and shows fluctuation).

**Figure 12:** Training progress of adam of ResNet without image processing (this depicts the training progress of adam and ResNet before the image processing phase and shows fluctuation).

**Figure 13:** Training progress of RMSPROP of ResNet without image processing (this depicts the training progress of rmsprop and ResNet before the image processing phase and shows fluctuation).

**Figure 14:** Training progress of SGDM and AlexNet after image processing (this depicts the training progress of SGDM and ResNet after the image processing phase and shows no fluctuation in the end and smoothes the training curve).

**Table 1:** Limitations of previous studies (it explains the results of previous studies and shows the previous studies research gap).

Publications	Methods	Datasets	Accuracy (%)	Limitations
Pansombut et al. [35]	CNN	Image (public)	80	(i) Low-ratio dataset
				(ii) Data image processing layer

Madhukar et al. [34]	SVM	Image (public)	93.5	(i) Low-ratio dataset
				(ii) Minor image classes
				(iii) Data image processing layer

Supardi et al. [33]	KNN	Image (public)	86	(i) Low-ratio dataset
				(ii) Data image processing layer

Patel and Mishra [32]	SVM	Image (public)	93.57	(i) Data image processing layer

Laosai and Chamnongthai [31]	SVM	Image (public)	92	(i) Low-ratio dataset
				(ii) Data image processing layer

Faivdullah et al. [30]	SVM	Feature (public)	79.38	(i) Required handcrafted features

Setiawan et al. [29]	SVM, K-means	Image (public)	87	(i) Low-diverse dataset
				(ii) Low-ratio dataset
				(iii) Data image processing layer

Kumar et al. [28]	KNN, Naïve Bayes, CNN	Image (public)	92.8	(i) Low-ratio dataset
				(ii) Less number of classes

Loey et al. [27]	CNN, AlexNet	Image (public)	94.3	(i) Low-ratio dataset
				(ii) Data image processing
				(iii) Less number of classes

**Table 2:** Pseudocode of the proposed model (this depicts the algorithm of the current study and research methodology from data fetching to training and testing and also it explains every training model).

Steps	Codes
1	Input cancerous white blood cell images
2	Image preprocessing
3	Data division into training and testing
4	Store into cloud (*£*)
5	Input training images to deep learning algorithms

6	AlexNet
	1- SGDM
	2- Adaptive moment (ADAM)
	3- Root mean square propagation (RMSPROP)
	Check learning criteria
	**If** meet
	Store into private cloud
	**Else** applying image preprocessing
	Input image preprocessed images to deep learning algorithm
	AlexNet
	4- SGDM
	5- ADAM
	6- RMSPROP
	Check learning criteria
	**If** meet
	Store into private cloud
	**Else**
	Retrain

7	ResNet
	1- SGDM
	2- ADAM
	3- RMSPROP
	Check learning criteria
	**If** meet
	Store into private cloud
	**Else** applying image preprocessing
	Input image preprocessed images to deep learning algorithm
	ResNet
	4- SGDM
	5- ADAM
	6- RMSPROP
	Check learning criteria
	**If** meet
	Store into private cloud
	**Else**
	Retrain

8	ResNet
	1- SGDM
	2- ADAM
	3- RMSPROP
	Check learning criteria
	**If** meet
	Store into private cloud
	**Else** applying image preprocessing
	Input image preprocessed images to deep learning algorithm
	ResNet
	4- SGDM
	5- ADAM
	6- RMSPROP
	Check learning criteria
	**If** meet
	Store into private cloud
	**Else**
	Retrain

9	Access all private cloud
	Check the learning criteria of the best deep learning trained models
	**If** meet
	Select semi-best model and store it in other private cloud
	**Else**
	Retry

10	Import one best trained model
11	Input pre-processed test images
12	Test analysis
13	Applying statistical performance matrix

The article "Hematologic Cancer Detection Using White Blood Cancerous Cells Empowered with Transfer Learning and Image Processing" was published in 2023. Journal: J Healthc Eng.

**Table 3:** AlexNet training results after image processing (this depicts the AlexNet training results of all learners after image processing).

AlexNet					
Model	Iterations	Learning rate (LR)	Epoch	Classification accuracy (%)	Missclassification rate (%)
SGD moment	5800	0.001	100	99.2	0.8
ADAM				95.31	4.69
RMSPROP				96.09	3.91

**Table 4:** Training results of ResNet models after image processing (this depicts the ResNet training results of all learners after image processing).

AlexNet					
Models	Iterations	Learning rate (LR)	Epoch	Classification accuracy (%)	Missclassification rate (%)
SGD moment	5800	0.001	100	68.75	31.25
ADAM				68.79	31.21
RMSPROP				69.53	30.47

**Table 5:** Training results of mobile net models after image processing (this depicts the mobile net training results of all learners after image processing).

AlexNet					
Models	Iterations	Learning rate (LR)	Epoch	Classification accuracy (%)	Missclassification rate (%)
SGD moment	5800	0.001	100	69.53	30.47
ADAM				72.3	27.7
RMSPROP				73.44	26.56

**Table 6:** AlexNet confusion matrix of testing samples after image processing (this depicts the testing confusion metric of AlexNet after image processing).

AlexNet			
Model (SGDM)	Lymphocyte	Monocyte	Neutrophil
Sample = 2238			

Lymphocyte	719	0	9
Monocyte	16	742	25
Neutrophil	10	1	716

AlexNet			
Model (ADAM)	Lymphocyte	Monocyte	Neutrophil
Sample = 2238			

Lymphocyte	674	15	14
Monocyte	22	703	16
Neutrophil	49	25	720

AlexNet			
Model (RMSPROP)	Lymphocyte	Monocyte	Neutrophil
Sample = 2238			

Lymphocyte	714	30	36
Monocyte	16	680	22
Neutrophil	15	33	692

The article "Hematologic Cancer Detection Using White Blood Cancerous Cells Empowered with Transfer Learning and Image Processing" was published in 2023. Journal: J Healthc Eng.

**Table 7:** Mobile net confusion matrix of testing samples after image processing (this depicts the testing confusion metric of the mobile net after image processing).

MobileNet			
Model (SGDM)	Lymphocyte	Monocyte	Neutrophil
Sample = 2238			

Lymphocyte	678	44	47
Monocyte	0	284	308
Neutrophil	67	415	388

MobileNet			
Model (ADAM)	Lymphocyte	Monocyte	Neutrophil
Sample = 2238			

Lymphocyte	676	3	5
Monocyte	28	339	348
Neutrophil	41	401	390

MobileNet			
Model (RMSPROP)	Lymphocyte	Monocyte	Neutrophil
Sample = 2238			

Lymphocyte	729	13	14
Monocyte	16	559	570
Neutrophil	0	171	159

**Table 8:** RESNET confusion matrix of testing samples after image processing (this depicts the testing confusion metric of ResNet after image processing).

ResNet			
Model (SGDM)	Lymphocyte	Monocyte	Neutrophil
Sample = 2238			

Lymphocyte	717	1	0
Monocyte	21	409	391
Neutrophil	7	333	352

ResNet			
Model (ADAM)	Lymphocyte	Monocyte	Neutrophil
Sample = 2238			

Lymphocyte	736	1	1
Monocyte	1	319	314
Neutrophil	8	423	428

ResNet			
Model (RMSPROP)	Lymphocyte	Monocyte	Neutrophil
Sample = 2238			

Lymphocyte	728	6	3
Monocyte	16	608	612
Neutrophil	1	129	128

**Table 9:** Statistical matrix test results of blood cancer prediction after image processing (this depicts the statistical results of all models performed in the current study).

*AlexNet*											
*Stochastic gradient descent moment (%)*											
CA	Sen	PPV	FPR	FNR	LPR	LNR	FMI	F1	NPV	Spec	MCR
97.3	96.51	98.76	0.60	3.49	160.10	0.04	97.63	97.62	98.28	99.40	2.7

*Adaptive moment estimation (%)*											
CA	Sen	PPV	FPR	FNR	LPR	LNR	FMI	F1	NPV	Spec	MCR
93.07	90.47	95.87	1.94	9.53	46.58	0.10	93.13	93.09	95.37	98.06	6.03

*Root mean square propagation (%)*											
CA	Sen	PPV	FPR	FNR	LPR	LNR	FMI	F1	NPV	Spec	MCR
93.02	95.84	91.54	4.42	4.16	21.68	0.04	93.66	93.64	97.87	95.58	6.08

*MobileNet*											
*Stochastic gradient descent moment (%)*											
CA	Sen	PPV	FPR	FNR	LPR	LNR	FMI	F1	NPV	Spec	MCR
60.5	91.01	88.77	6.12	8.99	14.86	0.10	89.58	89.56	95.42	93.88	39.5

*Adaptive moment estimation (%)*											
CA	Sen	PPV	FPR	FNR	LPR	LNR	FMI	F1	NPV	Spec	MCR
63.0	90.74	98.83	0.54	9.26	46.55	0.09	94.70	94.61	95.42	99.46	37.0

*Root mean square propagation (%)*											
CA	Sen	PPV	FPR	FNR	LPR	LNR	FMI	F1	NPV	Spec	MCR
64.09	97.85	96.43	1.82	2.15	53.86	0.02	97.14	97.14	98.92	98.18	35.01

*ResNet*											
*Stochastic gradient descent moment (%)*											
CA	Sen	PPV	FPR	FNR	LPR	LNR	FMI	F1	NPV	Spec	MCR
66.2	96.24	99.86	0.07	3.76	30.15	0.04	98.03	98.02	98.92	99.93	83.8

*Adaptive moment estimation (%)*											
CA	Sen	PPV	FPR	FNR	LPR	LNR	FMI	F1	NPV	Spec	MCR
66.5	59.55	88.04	6.31	40.45	9.43	0.43	72.40	71.04	98.92	93.69	33.5

*Root mean square propagation (%)*											
CA	Sen	PPV	FPR	FNR	LPR	LNR	FMI	F1	NPV	Spec	MCR
65.6	59.28	87.92	6.34	40.72	9.35	0.43	72.20	70.82	98.92	93.66	34.4

The article "Hematologic Cancer Detection Using White Blood Cancerous Cells Empowered with Transfer Learning and Image Processing" was published in 2023. Journal: J Healthc Eng.

**Table 10:** Testing results before image processing (this depicts the comparative results of all models like classification accuracy and miss-classification rate).

Models	CA (%)	MCR (%)
*AlexNet*		
SGDM	78.6	21.4
ADAM	74.3	25.7
RMSPORP	68.3	31.7

*ResNet*		
SGDM	71.0	29.0
ADAM	75.0	25.0
RMSPROP	56.0	44.0

*MobileNet*		
SGDM	63.1	36.9
ADAM	73.8	26.2
RMSPROP	60.9	39.1

**Table 11:** Comparative analysis with previous studies (this depicts the comparative study of current research with previous research).

Publication	Image processing	Model	Dataset	Accuracy (%)	MCR (%)
Pansombut et al. [35]	No	CNN	Image (public)	80	20
Madhukar et al. [34]	No	SVM	Image (public)	93.5	6.5
Supardi et al. [33]	No	KNN	Image (public)	86	14
Patel and Mishra [32]	No	SVM	Image (public)	93.57	6.53
Laosai and Chamnongthai [31]	No	SVM	Image (public)	92	18
Faivdullah et al. [30]	No	SVM	Feature (public)	79.38	20.72
Setiawan et al. [29]	No	SVM, K-means	Image (public)	87	13
Kumar et al. [28]	No	KNN, Naïve Bayes, CNN	Image (public)	92.8	17.2
Loey et al. [27]	No	CNN, AlexNet	Image (public)	94.3	5.7
The proposed model	Yes	Transfer learning (AlexNet, ResNet, MobileNet)	Image (public, 10,000 instances)	97.3	2.7

## Data Availability

The data used in this paper can be requested from the corresponding author upon request.

## Abbreviations

SVM: Support vector machine
CNN: Convolutional neural network
KNN: K-nearest neighbor
WBC: White blood cells
SGD: Stochastic gradient descent
CA: Classification accuracy
NPV: Negative predicted value
MCR: Miss-classification rate
PPV: Positive predicted value
LPR: Likelihood positive ratio
LNR: Likelihood negative ratio
FNR: False negative rate
FPR: False positive rate
FMI: Fowlkes mallows index
ADAM: Adaptive moment estimation
RMSPROP: Root mean square propagation
ANOVA: Analysis of variance.
